The article "Differentially Private Singular Value Decomposition for Training Support Vector Machines" was retracted in 2023. Reasons: unreliable results or conclusions; concerns about the data; concerns about the results or conclusions; concerns about the peer review.

# Differentially Private Singular Value Decomposition for Training Support Vector Machines

**DOI:** 10.1155/2022/2935975

**Published:** 2022-03-26

**Authors:** Zhenlong Sun, Jing Yang, Xiaoye Li

**Affiliations:** ^1^College of Computer Science and Technology, Harbin Engineering University, Harbin 150001, China; ^2^College of Computer and Control Engineering, Qiqihar University, Qiqihar 161006, China

## Abstract

Support vector machine (SVM) is an efficient classification method in machine learning. The traditional classification model of SVMs may pose a great threat to personal privacy, when sensitive information is included in the training datasets. Principal component analysis (PCA) can project instances into a low-dimensional subspace while capturing the variance of the matrix *A* as much as possible. There are two common algorithms that PCA uses to perform the principal component analysis, eigenvalue decomposition (EVD) and singular value decomposition (SVD). The main advantage of SVD compared with EVD is that it does not need to compute the matrix of covariance. This study presents a new differentially private SVD algorithm (DPSVD) to prevent the privacy leak of SVM classifiers. The DPSVD generates a set of private singular vectors that the projected instances in the singular subspace can be directly used to train SVM while not disclosing privacy of the original instances. After proving that the DPSVD satisfies differential privacy in theory, several experiments were carried out. The experimental results confirm that our method achieved higher accuracy and better stability on different real datasets, compared with other existing private PCA algorithms used to train SVM.

## 1. Introduction

In the past decade, more and more personal information has been stored in electronic databases for machine learning and personalized recommendation. The data sharing and analysis bring lots of convenience to people's lives, but pose a great threat to personal privacy. Support vector machine (SVM) [1] is a popular classification method that searches for the best hyperplane that separates two class instances by solving a quadratic optimization problem. It has been applied in pattern recognition such as image recognition and text classification. In the classification model of SVM, the most serious privacy issue is that the support vectors (SVs) are directly obtained from the training datasets [2]. Therefore, the classification model should be privately published to avoid disclosing personal sensitive information.

Differential privacy (DP) [3–6] has a strict mathematical definition and the level of privacy protection can be quantified by a small parameter *ɛ* named privacy budget. DP has been becoming an accept standard. It guarantees that the result of an analysis is virtually independent of the addition or removal of one record. DP has attracted a growing research attention [7]. The common mechanisms for implementing DP include Laplace mechanism [8], Gaussian mechanism [9], and exponential mechanism [10].

The article "Differentially Private Singular Value Decomposition for Training Support Vector Machines" was retracted in 2023. Reasons: unreliable results or conclusions; concerns about the data; concerns about the results or conclusions; concerns about the peer review.

Principal component analysis (PCA) [9] solves a low-rank subspace, which completely captures the variance of matrix *A*. The main advantages of working with the low-rank approximation of *A* include higher time and space efficiency, less noise, and removal of correlation between features. Through PCA, the original instances are projected into a low-dimensional subspace and the features become linearly independent. Eigenvalue decomposition (EVD) and singular value decomposition (SVD) are two common algorithms to perform PCA. They are related to the familiar theory of matrix diagonalization. The EVD is used for a symmetric matrix and SVD for an arbitrary matrix. Furthermore, SVD does not need to compute the matrix of covariance compared with EVD [11].

This study researches the privacy leakage problem of SVM classifier. To overcome some shortcomings in the existing private SVMs, a differentially private singular value decomposition (DPSVD) algorithm is proposed to keep SVs private in the classification model of SVM. This study makes the following innovations:

- The authors proposed an idea that projecting the training instances into the low-dimensional singular subspace and the SVM can train the classification model on it while not violating the privacy requirements for the training data.
- The projection process of the DPSVD satisfies DP, and the generated singular vectors are also private which can be provided directly to users for classification testing.
- In the DPSVD, the projection process is implemented by SVD. The main advantage is that SVD does not need to calculate the matrix of covariance compared with EVD. It takes up a lot of memory space for high-dimensional data.
- Our method protects privacy of the training instances before training the classification model; many optimization methods of SVMs can be applied directly to the training progress.
- After proving that the DPSVD satisfies differential privacy in theory, several experiments were carried out. The experimental results confirm that our method achieved higher accuracy and better stability on different real datasets, compared with other existing private PCA algorithms used to train SVM.

## 2. Related Work

From a privacy perspective, SVMs have serious privacy issues, because SVs tend to be directly obtained from the training datasets. There is a lot of work to solve this privacy problem based on DP. Chaudhuri et al. [12, 13] proposed two perturbation-based methods for problems like linear SVM classification. For nonlinear kernel SVM, they derived the kernel function through random projection and linearized the function. However, it is hard to analyze the sensitivity of the output perturbation, and the differentiability criteria are required in the loss function of objective perturbation. To learn SVM privately, Rubinstein et al. [14] developed two feature mapping methods by adding noise to the output classifier. But their methods only apply to the kernels that do not change with translation. Li et al. [15] designed a mixed SVM, which alleviate much of the noise through Fourier transform based on a few open-consented information. Zhang et al. [16] proposed DPSVMDVP by adding Laplace noise to the dual variables based on the error rate. Liu et al. [17] presented an innovative private classifier called LabSam by random sampling under the exponential mechanism. Sun et al. [18] proposed the DPWSS, which introduces randomness into SVM training; they also proposed another private SVM algorithm DPKSVMEL based on exponential and Laplace hybrid mechanism [19] for the kernel SVM to prevent privacy leakage of the SVs.

The article "Differentially Private Singular Value Decomposition for Training Support Vector Machines" was retracted in 2023. Reasons: unreliable results or conclusions; concerns about the data; concerns about the results or conclusions; concerns about the peer review.

PCA constructs a set of new features to describe the instances in a low-dimensional subspace. When the generated projection vectors are private, the new instances in the low-dimensional subspace are private as well, and they can be used directly to train SVMs without compromising the privacy of the instances. There are several researches on private PCA. Blum et al. [20] developed SuLQ by disturbing the matrix of covariance with Gaussian noise. However, the greatest eigenvalue might be not real, due to the asymmetry of the noise matrix. Chaudhuri et al. [21] modified SuLQ framework with a symmetric noise matrix and used it for data publishing. Dwork et al. [9] disturbed the matrix of covariance with Gaussian noise. Imtiaz and Sarwate [22, 23] and Jiang et al. [24] disturbed the matrix of covariance with Wishart noise and it guarantees that the perturbed matrix of covariance is positive semidefinite. Xu et al. [25] and Huang et al. [26] added symmetric Laplace noise to the matrix of covariance. Those methods above all generate the perturbed matrix of covariance by adding a noise matrix and then perform EVD to implement PCA. And only [26] measured the availability of the private PCA by SVM, but not to research private PCA from the privacy perspective of SVM. Recently, SVD has been widely used in collaborative filtering [27], deep learning [28], data compression [29, 30], and images watermarking [31]. There are few researches on privacy-preserving data mining based on SVD. Keyvanpour et al. [32] defined a method that combined SVD and feature selection to benefit from the advantages of both domains. Li et al. [33] gave a new algorithm for protecting privacy based on nonnegative matrix factorization and SVD. Kousika et al. [34] proposed a methodology based on SVD and 3D rotation data perturbation for preserving privacy of data.

The article "Differentially Private Singular Value Decomposition for Training Support Vector Machines" was retracted in 2023. Reasons: unreliable results or conclusions; concerns about the data; concerns about the results or conclusions; concerns about the peer review.

## 3. Background

Table 1 summarizes the symbols used in this study.

### 3.1. Support Vector Machines

Given training instances *x*_*i*_ ∈ *R*^*d*^ and labels *y*_*i*_ ∈ {1, −1} the classification model of SVM can be obtained by solving the following optimization problem [35]:

(1) $$\begin{array}{c} \underset{\alpha }{\min}f\left(\alpha \right)=\frac{1}{2}\alpha^{T}Q\alpha -e^{T}\alpha . \end{array}$$

(2) $$\begin{array}{c} \text{Subject to}\;0\leq \alpha_{i}\leq C,i=1,...,l \end{array}$$

where ***α*** is a dual vector; *Q* is a symmetric matrix, *Q*_*ij*_ = *y*_*i*_*y*_*j*_*K*(*x*_*i*_, *x*_*j*_), and *K* is the kernel function.

Let *x* be a new instance. The label of *x* can be predicted by the decision function as follows:

(3) $$\begin{array}{c} f\left(x\right)=\sum_{i=1}^{n}\alpha_{i}y_{i}K\left(x_{i},x\right)+b. \end{array}$$

In the classification model, only the SVs determine the maximal margin and correspond to the nonzero *α*_*i*_s, and others equal zero. From a privacy perspective, the classification model has serious privacy issues as the SVs are intact instances.

### 3.2. Principal Component Analysis

PCA computes a low-rank subspace and achieves the dimensionality reduction for high-dimensional data, shedding light on the use of private SVM in high-dimensional data classification. For a given data matrix *D* ∈ *R*^*n*×*d*^ with *d* features of *n* instances, the *i*-th row of *D* is denoted by *x*_*i*_ and assumes that its *ℓ*_2_ norm satisfies ||*x*_*i*_||_2_ ≤ 1. After the matrix is centralized by column, the matrix of covariance can be obtained as

(4) $$\begin{array}{c} A=\frac{1}{n}D^{T}D=\frac{1}{n}\sum_{i=1}^{n}x_{i}^{T}x_{i}. \end{array}$$

The matrix of covariance is a real symmetric matrix; therefore its eigenvalues and corresponding eigenvectors can be obtained by EVD:

(5) $$\begin{array}{c} Av_{i}=\lambda_{i}v_{i}, \end{array}$$

where *λ*_*i*_ is one of the eigenvalues and *v*_*i*_ is its corresponding eigenvector. The *λ*_*i*_ could be treated as variance of the *i*-th principal component to denote its importance and is sorted in descending order. Generally, the threshold of the accumulative contribution rate of principal components *γ* (0 ≤ *γ* ≤ 1) is set to decide the target dimension *k* by

(6) $$\begin{array}{c} \frac{\sum_{\mathrm{i=1}}^{k}\lambda_{i}}{\sum_{\mathrm{i=1}}^{d}\lambda_{i}}\geq \gamma . \end{array}$$

According to the diagonalization theory of matrix and (5), it obtains another representation of EVD as follows:

(7) $$\begin{array}{c} A=V\sum V^{T}, \end{array}$$

where *V* is an orthogonal matrix consisting of eigenvectors in columns and *∑* is a diagonal matrix taking eigenvalues as diagonal entries. Compared with EVD, SVD can be applied to an arbitrary real matrix and it does not need to calculate matrix of covariance. The representation of SVD is shown as follows:

(8) $$\begin{array}{c} D=USV^{T}, \end{array}$$

where *U* and *V* are the left and right singular matrices, which consist of left and right singular vectors, respectively; *S* is a diagonal matrix taking singular values as diagonal entries. The singular value *σ*_*i*_ is also sorted in descending order. The relationship between EVD and SVD is as follows:

(9) $$\begin{array}{c} A=\frac{1}{n}D^{T}D=\frac{1}{n}{\left(USV^{T}\right)}^{T}\left(USV^{T}\right)=\frac{1}{n}VSU^{T}USV^{T}=\frac{1}{n}VSSV^{T}=\frac{1}{n}VS^{2}V^{T}, \end{array}$$

(10) $$\begin{array}{c} \tilde{A}=\frac{1}{n}DD^{T}=\frac{1}{n}\left(USV^{T}\right){\left(USV^{T}\right)}^{T}=\frac{1}{n}USV^{T}VSU^{T}=\frac{1}{n}USSU^{T}=\frac{1}{n}US^{2}U^{T}, \end{array}$$

where *U*^*T*^*U*=*I* and *V*^*T*^*V*=*I*, because *U* and *V* are both made up of unit orthogonal vectors; they also are called orthonormal basis matrices. The coefficient 1/*n* has nothing to do with the eigenvectors and the proportionality of eigenvalues. We generally use *D*^*T*^*D* to approximate the matrix of covariance. From (9) and (10), we can conclude that the SVD of an arbitrary real matrix yields a similar result to the EVD of its matrix of covariance. In the SVD of *D*, the right singular vectors serve as the eigenvectors of *D*^*T*^*D*, and the left ones serve as those of *DD*^*T*^. The singular values equal the square roots of the nonzero eigenvalues of *D*^*T*^*D* and *DD*^*T*^.

The article "Differentially Private Singular Value Decomposition for Training Support Vector Machines" was retracted in 2023. Reasons: unreliable results or conclusions; concerns about the data; concerns about the results or conclusions; concerns about the peer review.

### 3.3. Differential Privacy

**Definition 1 .**

(differential privacy (see [3])). A stochastic mechanism *M* satisfies (*ε*, *δ*)-differential privacy, provided that, for every two adjacent matrices *D* and *D′* differing in exactly one row, and for all subsets of probable outcomes *O*⊆ Range(*M*),

(11) $$\begin{array}{c} \mathrm{Pr}\left[M\left(D\right)\in O\right]\leq \;\exp\left(\varepsilon \right)\times \mathrm{Pr}\left[M\left(D^{\prime }\right)\in O\right]+\delta . \end{array}$$

When *δ* equals zero, *M* satisfies *ε*-differential privacy.

**Definition 2 .**

(sensitivity (see [3])). For a given function *q* : *D*⟶*R*^*d*^, and adjacent matrices *D* and *D′*, the sensitivities *S*_*1*_ and *S*_*2*_ of function *q* can be, respectively, expressed as

(12) $$\begin{array}{c} S_{1}=\underset{D,D^{\prime }}{\max}{\left\|q\left(D\right)-q\left(D^{\prime }\right)\right\|}_{1}\text{ and }S_{2}=\underset{D,D^{\prime }}{\max}{\left\|q\left(D\right)-q\left(D^{\prime }\right)\right\|}_{2}. \end{array}$$

*S*_*1*_ corresponding to *ℓ*_1_ norm is usually used in Laplace mechanism, while *S*_*2*_ corresponding to *ℓ*_2_ norm is used in Gaussian mechanism.

**Definition 3 .**

(Laplace mechanism (see [8])). For a numeric function *q* : *D*⟶*R*^*d*^, with scale factor *b* = *S*_*1*_/*ɛ*. The Laplace mechanism, which adds independent random noise distributed as *Laplace*(*b*) to each output of *q*(*D*), ensures *ε*-differential privacy.

**Definition 4 .**

(Gaussian mechanism (see [9])). For a numeric function *q* : *D*⟶*R*^*d*^, let $\beta =S_{2}\sqrt{2\;\ln\left(1.25/\delta \right)}/\varepsilon$. The Gaussian mechanism, which adds independent random noise distributed as *N*(0, *β*^*2*^) to each output of *q*(*D*), ensures (*ε*, *δ*)-differential privacy.

## 4. Materials and Methods

To overcome the shortcomings in the existing private SVMs, we proposed the DPSVD. The DPSVD privately projects the original instances to a low-dimension singular subspace and trains a SVM classification model in it to protect the privacy of training instances.

### 4.1. Algorithm Description: Algorithm 1 Is the Pseudocode of the DPSVD

The algorithm 1 describes the implementation process of the DPSVD for training a private classification model of SVM. Firstly, it generates a noise matrix sampled from Gaussian distribution, and this step does not need to symmetrize the noise matrix as the existing private PCA algorithms. Secondly, it adds the noise matrix to the raw data matrix rather than the matrix of covariance of the raw data. When features far outnumber instances, the matrix of covariance will take up a lot of memory space, especially for high-dimensional data. Meanwhile, the matrix of covariance will magnify errors in the raw data to some extent. Thirdly, the DPVSD algorithm computes the singular values and singular matrices by SVD, while the existing private PCA algorithms use EVD. Generally, SVD can be considered a black box and has higher execution efficiency compared with EVD, although the two decomposition methods generate the same projection subspace by singular vectors or eigenvectors under the nonprivate situation. There are similar computing processes with the EVD in the next three steps. Lastly, the DPSVD distributes the private classification model to predict the new instances, prior to idea that it projects them to the same singular subspace by the private singular vectors. In brief, the DPSVD trains a private SVM classifier for predicting the new instances in future.

The article "Differentially Private Singular Value Decomposition for Training Support Vector Machines" was retracted in 2023. Reasons: unreliable results or conclusions; concerns about the data; concerns about the results or conclusions; concerns about the peer review.

### 4.2. Privacy Analysis

Firstly, the sensitivity of the function *q*(*D*) is analyzed, and then the DPSVD is demonstrated to satisfy (*ε*, *δ*)-differential privacy. In the DPSVD algorithm, the noise matrix is added to the data matrix *D*; therefore *q*(*D*) = *D*. Given that two adjacent data matrices *D* and *D′* differ by exactly one row corresponding to an instance, we set *D′* obtained from *D* by deleting the last row, *D*=[*x*_1_, ..., *x*_*n*_]^*T*^ ∈ *R*^*n*×*d*^ and *D*′=[*x*_1_, ..., *x*_*n*−1_]^*T*^ ∈ *R*^(*n* − 1)×*d*^, and assume each row has unit *ℓ*_2_ norm ||*x*_*i*_||_2_≤1 at the most.

**Lemma 1 .**

The sensitivity of the function *q*(*D*) *S*_2_ equals one.

**Proof**

According to Definition 2, it obtains *S*_2_ by the following inequation:

(13) $$\begin{array}{c} S_{2}=\underset{D,D^{\prime }}{\max}{\left\|q\left(D\right)-q\left(D^{\prime }\right)\right\|}_{2}=\underset{D,D^{\prime }}{\max}{\left\|D-D^{\prime }\right\|}_{2}=\underset{D,D^{\prime }}{\max}{\left\|x_{n}\right\|}_{2}\leq 1 \end{array}$$

Therefore, the sensitivity of the function *q*(*D*) equals one.

**Theorem 1 .**

The DPSVD satisfies (*ε*, *δ*)-differential privacy.

**Proof**

To demonstrate that the DPSVD satisfies (*ε*, *δ*)-differential privacy, it is necessary to demonstrate every step in the algorithm satisfies it. According to Lemma 1, it obtains that *S*_2_ equals one. Let $\beta =S_{2}\sqrt{2\;\ln\left(1.25/\delta \right)}/\varepsilon =\sqrt{2\;\ln\left(1.25/\delta \right)}/\varepsilon$; then Step (1) and Step (2) satisfy DP according to Definition 4. Step (3) and Step (4) postprocess the private data matrix *D′*; they also satisfy DP. Step (5) generates the private singular vectors *V*_*k*_; the projected instances *Y* in the low-dimensional singular subspace are private as well. Meanwhile, *Y* does not need to be distributed to users. Step (6) and Step (7) compute the classification model based on private projection instances and distribute it together with private singular vector to predict the new instances. The last three steps do not violate the privacy requirement of DP. Therefore, the DPSVD satisfies (*ε*, *δ*)-differential privacy.

### 4.3. Algorithm Comparison

The three algorithms were compared theoretically between DPSVD, AG [9], and DPPCA-SVM [26] summarized in Table 2. Other ones have been compared by the DPPCA-SVM algorithm. Our algorithm uses SVD to perform PCA; it does not need to compute matrix of covariance and symmetrize the noise matrix as the description above. It obtains the same noise scale as AG algorithm, because they use identical mechanism of DP to generate the noise matrix.

The article "Differentially Private Singular Value Decomposition for Training Support Vector Machines" was retracted in 2023. Reasons: unreliable results or conclusions; concerns about the data; concerns about the results or conclusions; concerns about the peer review.

Therefore, the classification model and the singular vectors for projection are both private; they can be used to predict the new instances in the same singular subspace. The main advantage of the DPSVD compared with other private SVMs is that our algorithm trains the classification model in the private low-dimensional singular subspace generated by SVD. In this way, the features of the instances in the singular subspace become linearly independent and low-dimensional and therefore have higher time and space efficiency for training the classification model. The difference between our algorithm with other private PCA algorithms is that it does not need to calculate the matrix of covariance or symmetrize the noise matrix. Meanwhile, the DPSVD protects privacy of the training instances before training the classification model; many optimization methods of SVMs can be applied directly to the training progress.

## 5. Results

### 5.1. Datasets

Our experiments were carried out on four popular datasets for testing SVM performance.  Table 3 describes their basic information, including the number of the instances, the number of the features, and the ranges of values in the data. They are accessible at https://www.csie.ntu.edu.tw/∼cjlin/libsvmtools/datasets/ and http://archive.ics.uci.edu/ml/datasets.php. It trains the SVM to compare the performance of algorithms based on LIBSVM (version 3.25) [36] with the radial basis function as the kernel function and default parameters.

### 5.2. Algorithm Performance Experiments

The performance of the DPSVD was compared with AG, DPPCA-SVM, and the nonprivate SVM on the four real datasets. In the experiments, it designed two metrics of algorithm performance *Accuracy* and *SV*. *Accuracy* denotes how accurate the classification is, and *SV* denotes how many SVs are contained in the classifier. The higher the *Accuracy*, the greater the usability of the classifier. The closer *SV* to that of nonprivate SVM, the better the stability of the algorithm. The privacy budget *ɛ* was set at 0.1, 0.5, and 1, *δ* at 1/*n*^2^, and the accumulative contribution rate of principal components *γ* at 90%. Three private algorithms were implemented five times under every privacy budget parameter. The mean values, standard deviation, and maximum and minimum values of the two metrics are given in Table 4.

From the experiments results in Table 4, the DPSVD was the most accurate in classification than the other two private classifiers under different privacy budget for most of the datasets. Sometimes, our algorithm even outperformed the nonprivate SVM. This is mainly because our algorithm removes the linear dependence between features and unimportant features by SVD. Meanwhile, our algorithm has the better stability of the algorithm as its *SV* is much closer to the nonprivate SVM. To compare algorithm performance more intuitively, the mean values of the two metrics for the four algorithms are shown in Figures 1–8.

The article "Differentially Private Singular Value Decomposition for Training Support Vector Machines" was retracted in 2023. Reasons: unreliable results or conclusions; concerns about the data; concerns about the results or conclusions; concerns about the peer review.

In Figure 1 to Figure 3, the DPSVD achieved the highest classification accuracy in the three private algorithms and closer to the nonprivate SVM than the other two algorithms. In Figure 4, the AG achieved the higher classification accuracy than the DPSVD as the privacy budget increases. In Figure 5 to Figure 8, the DPSVD contained the closer number of SVs in the classifier to the nonprivate SVM than the other two algorithms. Therefore, the PDSVD achieved higher classification accuracy and better algorithm stability on most of the datasets and approximated the performance of the nonprivate SVM. The AG algorithm on dataset Musk in Figure 3 and the DPPCA-SVM algorithm on dataset Splice in Figure 4 have relatively lower classification accuracy. It also shows that the DPSVD has better algorithm stability.

## 6. Conclusions

To solve the privacy leak of SVM classifiers, especially on high-dimensional data, the DPSVD algorithm was proposed to project the training instances into the low-dimensional singular subspace and train a private SVM classifier on it while not violating the privacy requirements for the training data. The DPSVD is proved to satisfy DP. The main advantages of the DPSVD include three aspects. Firstly, it trains the classification model in the private low-dimensional singular subspace; therefore it has higher time and space efficiency compared with other private SVMs. Secondly, it does not need to calculate the matrix of covariance or symmetrize the noise matrix and has higher classification accuracy and better stability of the algorithm than other existing private PCA algorithms through the comparison experiments. Thirdly, it protects privacy of the training instances before training the classification model, and many optimization methods of SVMs can be applied directly to the training progress. Meanwhile, its algorithmic ideas can be applied to other machine learning areas to solve data privacy problems. However, the DPSVD can only solve the linear dependence between the data features. In future work, we will consider the nonlinear dependence to train a private classification model. In addition, the problem of data instances compression through SVD is another research direction.

## Figures and Tables

**Figure 1:** *Accuracy* at various *ɛ* on dataset A1a.

The article "Differentially Private Singular Value Decomposition for Training Support Vector Machines" was retracted in 2023. Reasons: unreliable results or conclusions; concerns about the data; concerns about the results or conclusions; concerns about the peer review.

**Figure 2:** *Accuracy* at various *ɛ* on dataset Mushrooms.

**Figure 3:** *Accuracy* at various *ɛ* on dataset Musk.

**Figure 4:** *Accuracy* at various *ɛ* on dataset Splice.

**Figure 5:** *SV* at various *ɛ* on dataset A1a.

**Figure 6:** *SV* at various *ɛ* on dataset Mushrooms.

**Figure 7:** *SV* at various *ɛ* on dataset Musk.

**Figure 8:** *SV* at various *ɛ* on dataset Splice.

**Algorithm 1:** DPSVD.

**Table 1:** Symbols.

Symbol	Description
*D*, *D′*	The adjacent matrix of datasets
*A*, $\tilde{A}$	Matrix of covariance
*x*_*i*_ ∈ *R*^*d*^.	Train instance
*y*_*i*_ ∈ {1, −1}.	Label
Α	Dual vector
*Q*	Symmetric matrix for kernel function
*K*	Kernel function
*E*	Vector composed entirely of ones
*C*	Upper limit of *α*
*λ*_*i*_	Eigenvalue
*v*_*i*_.	Eigenvector
Γ	The accumulative contribution rate of principal components
*U*, *V*	The singular vectors or eigenvectors matrix
*∑*, *S*	The singular values or eigenvalues diagonal matrix
*σ*_*i*_	Singular value
*I*	Unit diagonal matrix
*M*	A randomized mechanism
*O*	All subsets of possible outcomes of mechanism *M*
*ɛ*	Privacy budget
*β, δ*	Privacy parameter
*S*_*1*_, *S*_*2*_	The *ℓ*_1_ and *ℓ*_2_ sensitivity of function
*Laplace*(*b*)	Laplace noise (mean: 0; scale: *b*)
*N*(0, *τ*^*2*^)	Gaussian noise with (mean: 0; deviation: *τ*)

**Table 2:** The comparison between the three algorithms.

Algorithm	PCA	Adding mode	Noise form	Noise scale	Mechanism	Privacy level
DPSVD	SVD	*D*	Asymmetric	$O\left(\sqrt{d}/n\varepsilon \right)$	Gaussian	(*ε*, *δ*)
AG	EVD	*D* ^*T*^ *D/n*	Symmetric	$O\left(\sqrt{d}/n\varepsilon \right)$	Gaussian	(*ε*, *δ*)
DPPCA-SVM	EVD	*D* ^*T*^ *D/n*	Symmetric	*O*(*d*/*nε*)	Laplace	(*ε*, 0)

**Table 3:** Test datasets.

Indices	Datasets	Instances	Features	Ranges
1	A1a	1605	119	[0, 1]
2	Mushrooms	8124	112	[-1, 1]
3	Musk	6598	166	[-1, 1]
4	Splice	1000	60	[-1, 1]

**Table 4:** Performance comparison of algorithms on different datasets.

Datasets	*ɛ*	Algorithm	*Accuracy*				*SV*			
			Mean	Std	Max	Min	Mean	Std	Max	Min
A1a	--	SVM	83.49	--	--	--	754	--	--	--
	0.1	DPSVD	**83.35**	0.15	83.61	83.24	**763**	6	771	756
		AG	83.08	0.24	83.30	82.68	743	4	747	738
		DPPCA-SVM	82.58	0.58	83.30	81.93	771	12	783	754
	0.5	DPSVD	**83.50**	0.22	83.86	83.30	**755**	9	768	743
		AG	83.09	0.16	83.18	82.80	686	3	689	682
		DPPCA-SVM	83.07	0.50	83.49	82.24	764	14	778	747
	1	DPSVD	**83.59**	0.13	83.74	83.43	**753**	5	759	748
		AG	83.45	0.24	83.80	83.18	697	4	702	693
		DPPCA-SVM	83.46	0.41	84.11	82.99	756	14	778	742

Mushrooms	--	SVM	99.90	--	--	--	617	--	--	--
	0.1	DPSVD	**99.89**	0.01	99.90	99.88	**639**	39	700	607
		AG	99.18	0.02	99.21	99.15	518	3	521	514
		DPPCA-SVM	99.49	0.42	99.89	99.02	683	67	747	604
	0.5	DPSVD	**99.90**	0.01	99.90	99.89	**633**	25	674	607
		AG	99.19	0.05	99.26	99.14	524	5	531	517
		DPPCA-SVM	99.59	0.38	99.90	99.06	763	50	811	687
	1	DPSVD	**99.90**	0.00	99.90	99.90	**602**	26	625	559
		AG	99.79	0.04	99.83	99.73	445	22	469	417
		DPPCA-SVM	99.83	0.08	99.98	99.78	651	81	779	559

Musk	--	SVM	93.95	--	--	--	1351	--	--	--
	0.1	DPSVD	**94.08**	0.11	94.23	93.95	**1351**	15	1369	1330
		AG	88.96	0.08	89.09	88.89	1865	10	1876	1855
		DPPCA-SVM	93.97	0.20	94.23	93.74	1379	8	1391	1369
	0.5	DPSVD	**94.14**	0.11	94.27	94.00	**1359**	14	1379	1341
		AG	88.94	0.01	88.95	88.92	1866	6	1874	1858
		DPPCA-SVM	94.10	0.15	94.35	93.97	1336	15	1355	1315
	1	DPSVD	94.14	0.10	94.29	94.04	**1345**	10	1358	1333
		AG	88.93	0.02	88.95	88.91	1872	10	1887	1860
		DPPCA-SVM	**94.19**	0.17	94.35	93.92	1318	40	1384	1275

Splice	--	SVM	94.30	--	--	--	607	--	--	--
	0.1	DPSVD	**91.08**	0.75	92.40	90.60	635	17	662	616
		AG	90.56	0.83	91.30	89.30	**591**	16	605	568
		DPPCA-SVM	87.14	0.32	87.40	86.70	643	16	660	619
	0.5	DPSVD	92.00	0.80	92.80	90.70	**610**	10	625	600
		AG	**93.58**	0.38	94.00	93.00	588	5	595	582
		DPPCA-SVM	87.22	0.73	88.40	86.60	659	34	706	615
	1	DPSVD	92.36	0.56	93.10	91.80	**618**	19	645	594
		AG	**93.56**	0.31	93.90	93.10	594	3	599	591
		DPPCA-SVM	87.36	0.94	88.30	86.00	641	21	667	614

The article "Differentially Private Singular Value Decomposition for Training Support Vector Machines" was retracted in 2023. Reasons: unreliable results or conclusions; concerns about the data; concerns about the results or conclusions; concerns about the peer review.

## Data Availability

The raw data of the four datasets are available at https://www.csie.ntu.edu.tw/∼cjlin/libsvmtools/datasets/ and http://archive.ics.uci.edu/ml/datasets.php.
